# The Impact of Information and Communication Technologies (ICTs) on Health Outcomes: A Mediating Effect Analysis Based on Cross-National Panel Data

**DOI:** 10.1155/2022/2225723

**Published:** 2022-08-10

**Authors:** Mingxing Shao, Jing Fan, Zishan Huang, Mingyang Chen

**Affiliations:** International Business School, Beijing Foreign Studies University, Beijing, China

## Abstract

When ICTs (Information and Communications Technologies) are combined with healthcare, they can make a key contribution to gradually improve national health outcomes. The global outbreak of COVID-19 in 2020 further highlighted the important role of e-Health and m-Health service modes. This research structures a mediated effect model to explore dynamic relationships between ICT factors, ICT impacts, and national health outcomes, among which ICT factors are independent variables; ICT impacts are mediating variables, and national health outcome indicators selected from United Nations Millennium Development Goals (MDGs) and World Development Indicators are dependent variables. The fixed effect model is used to process a set of 141 countries' panel data from 2012 to 2016 from World Bank and World Economic Forum, while the classical three-step test method and Sobel test combined with fixed effects are used to test the mediated effects of the panel data. The results show that there are significant associations between ICT factors and national health outcome indicators, while only some of the partial mediated effects are proved. ICT environment and ICT usage can influence both the under-five mortality rate and adolescent fertility rate via ICT social impact. However, the mediated effect of ICT social impact on maternal mortality ratio and life expectancy at birth has not been confirmed. Meanwhile, the mediated effect of ICT economic impact has not been proven. This research is an interdisciplinary research in the field of information and communication technology and public health and reveals the path and mechanism whereby ICT factors improve national health outcomes, which can help global policymakers drive the next phase of the implementation of the Sustainable Development Goals (SDGs) and continue to improve the overall health at the national level.

## 1. Introduction

Using ICTs to efficiently provide services to citizens is an important area where digital technologies can make a difference in generating broad-based gains. ICT is an inclusive term, covering all communication equipment or application software: for example, radio, television, mobile phone, computer, network hardware and software, and satellite system, as well as various services and application software related to it, such as video conference and distance learning. The importance of ICTs is not the technology as such, but its enabling function in facilitating enhanced access to information and communication across large distances. ICTs have been used in many innovative ways to achieve social impacts, such as promoting access to basic services including health, finance, and insurance.

In the field of healthcare, key strategic applications of ICTs include e-Health and m-Health; E-Health and m-Health are increasingly employed—in combination with tools that build capacity and address the quality of care—to improve health systems, use resources efficiently, and plan for the progressive adoption of universal health coverage. Many people regard e-Health and m-Health as the next breakthrough in health system improvement, especially in developing nations. The integration of ICTs and healthcare can make a key contribution to improve lives and well-being worldwide and especially can assist the achievement of the health-related indicators of the United Nations Millennium Development Goals (MDGs). Take the COVID-19 outbreak in 2020 as an example, this emergency brought great challenges to all countries' medical and health system. In this fight against the pandemic, e-Health and m-Health service modes, represented by online telemedicine, showed their talents and played an important role.

ICTs are likely to fundamentally change the way public health is provided by influencing the economy and society. High-income countries have the capacity to increase investment in medical information and communication technologies to control and prevent child mortality and improve maternal health [1]. Developing countries may give priority to medical information technology projects in order to achieve rapid success, especially since the economic contraction will seriously hinder the implementation of online health policy [2]. This requires the introduction of more investment in ICT infrastructure to improve the availability and utilization of citizen broadband, so as to improve the penetration and application rate of e-Health and m-Health.

In academia, the previous studies on ICTs and health outcomes mostly stay at the conceptual or micro-level, or focus on the practical application of related technologies [3, 4], such as Blockchain technology in acquiring, managing, and sharing personal health information obtained from medical IoT (Internet of things) devices [5–8] or country-specific case studies or comparative studies [9–14]. Some studies have revealed positive relationships between ICTs and national health [1, 2, 15–17], which can confirm that ICTs ultimately improve national health outcomes by collecting and processing health information and enhancing communication and collaboration. However, through the literature review, we found that, on the one hand, the variables and dimensions used to measure ICTs in existing studies are not comprehensive; ICT factors are usually discussed as a whole and as one independent variable; on the other hand, most of the existing studies use cross-sectional data as the data resource, and there is a lack of consideration of the time dimension. Moreover, more importantly, the whole process and pathway of the effect of ICTs on the overall health level of the country are complex, and this issue has not been much explored in existing studies.

Based on the above discussion, this study explores the dynamic relationships between ICTs, the impact of ICTs, and the health levels of different countries over time. In this regard, two research questions are proposed to further explore this complex mechanism:

1. Do ICT factors influence the national health outcomes of a country over time?
2. What is the process and mechanism of ICT factors to improve national health outcomes?

In order to answer the above research questions, the panel data of 141 countries from 2012 to 2016 are taken as samples. ICT factors and ICT impact are extracted as independent variables and intermediary variables, respectively, from Networked Readiness Index (NRI) from the Global Information Technology Report. Four commonly used public health indicators are selected from MDGs and World Development Indicators as the explained variables. The classical stepwise regression method and Sobel test are used to test the mediated effects, so as to verify the mechanism of the relationships between the above variables.

The exploration of the above research questions is a useful addition and extension to the studies related to the impact and impact pathways of ICTs on national health outcomes. At the same time, answering these questions can help global policymakers to formulate health resource allocation and investment strategies, especially in the fields of healthcare and technology in developing countries, so as to achieve the best interests of people worldwide.

This paper is organized as follows: Section 2 discusses the literature review, Section 3 is regarding the research model and research hypothesis, Section 4 is the empirical research, Section 5 is the discussion, and Section 6 is the conclusion, limitation and future research.

## 2. Literature Review

### 2.1. Determinants of National Health Outcomes

The overall health of a country's population, or the national health outcomes of a country, is determined by multidimensional factors, including political, economic, social, and technological ones.

Politics has been found to have an impact on a country's national health outcomes. Multiple studies [18–20] discussed the relationship between political regimes and population health, finding that the level of democracy has a positive significance on population health. In particular, according to Patterson and Veenstra [20], electoral democracies are 11 years longer and 62.5% lower than other countries in terms of life expectancy and infant mortality rate, respectively. Based on an empirical analysis of India, Data [21] argued that political competition in the election can prompt the government to increase public health expenditure. Klomp and Haan [22] proposed that a higher degree of government stability usually brings about better health outcomes.

Various economic determinants of national health outcomes have been discussed in previous research. Granados [23] reviewed in detail the prior literature on the macroeconomic effects on mortality, particularly on the theory that mortality oscillates in a procyclical manner with the business cycle. Birgisdóttir and Ásgeirsdóttir [24] observed a statistically significant connection between economic recessions and a lower mortality rate in women aged 45–64. However, Burgard and Kalousova [25] suggested a weak link between the 2008 Financial Crisis and the decline of overall mortality in the US, despite an increase in suicide and mental distress among the affluent during this downturn. Apart from macroeconomic conditions, income and employment also contribute to population health. A global gradient was reported by Curran and Mahutga [26] in the association of income inequality with national health outcomes, featuring a stronger negative impact of income inequality on population health in poorer countries than in richer ones. Peckham et al. [27] discovered a relationship between employment quality and self-rated health, mental health, and occupational injury, and rendered material deprivation, employment-related stressors, and occupational risk factors the mediators between employment and health status. Employment has also been found to have an impact on maternal self-reported health [28].

Studies are rapidly emerging on social determinants of population health. Various forms of social inequality are believed to subject people to higher health risks. Clouston et al. [29] observed contributions of disparities in socioeconomic status (SES) and ethnicity to inequalities in colorectal cancer mortality, with people of lower SES as well as Black, Hispanic, and Asian races prone to higher mortality due to a dearth of age-appropriate medical testing and treatment. Cogburn [30] argued that cultural racism exacerbates multi-facet racial inequalities in health policy making, practice, and public reception. According to Harnois and Bastos [31], workplace mistreatment such as discrimination and harassment helps to shape the gender gap in workers' self-reported health. Besides, education is also a social determinant of health status, in particular of maternal–infant health status. Abreha and Zereyesus [32] pointed out a positive connection between women's empowerment by education and child health in Sub-Saharan Africa. Based on an empirical analysis of 153 countries from 1970 to 2016, Shorette and Burroway [33] found a distribution-specific advantage of women's education in reducing infant mortality; the significant impact is limited to the range of infant mortality rates from 11 to 55 deaths per 1000 live births.

Discussions over technological effects on population health lie primarily in ICT-health relations. Chauvin and Rispel [34] described the huge potential digital technologies possess to improve the health status of the mass public and health equity. Noh et al. [35] reported that mobile phones with a SIM card can lead to a substantial increase in the access to healthcare services for crisis-affected people in Afghanistan. Rafia et al. [36] confirmed ICTs' role in improving population health and longevity in Malaysia in both the short and long run. A systematic review is presented on the relationship between ICTs and health outcomes in the subsequent section.

### 2.2. ICTs and National Health Outcomes

Within the research of ICT factors and health outcomes, many multinational empirical studies have used similar indicators of national health development level. Mithas et al. [15], Wu [2] and Raghupathi [1] found that there is a positive correlation between ICTs and life expectancy. Mithas used a sample of 61 countries, and the other two samples are about 200 countries each. In addition, the authors studied the possible relationships between ICTs and mortality, fertility and *tuberculosis* in countries with different levels of development. Irawan and Koesoema [16] also found a significant relationship between ICTs, e-Health, child mortality and maternal health, mainly in developing countries, especially in sub-Saharan Africa, where maternal mortality still remains rather high; Mlambo et al. [37] proved that the use of ICTs can significantly reduce maternal mortality by enabling women' engagement in health treatment and welfare. Ahangama and Poo [17] found evidence of the moderating role of e-Health in improving infant survival in a sample of 55 countries.

All empirical studies use samples from countries with different levels of development, which may lead to some deviations. In the study of Wu [2] and Raghupathi [1], they isolated the developed countries and carried out a separate study and found that the positive correlation between ICT development and health outcomes was still widespread. The above authors tended to use the linear regression method, using cross-sectional data or panel data to test hypotheses. Tavares [38] also studied the relationship between ICTs, e-Health, and health outcomes in a sample of only 28 EU countries. Another innovation of the paper is that health outcomes are self-reported by individuals, rather than traditional population health indicators such as mortality or life expectancy.

In recent years, ICTs' role in health emergency response has garnered growing attention. Bajpai et al. [39] examined ICTs' performance in immediate relief and medical response in the context of COVID-19, including testing and diagnosis, patient-centric record keeping and case management, as well as telemedicine. Besides, ICTs are conducive to public mental health in the era of social distancing by helping people stay socially connected [40].

It is important to note that most of the studies focus on EU countries, while other regional or global studies account for a small proportion. This is due to the substantial sources of databases of the EU. Compared with WHO and the World Bank, EU indicators are more comprehensive, and most of them are numerical data, which is conducive to more complex data analysis.

### 2.3. ICT Impacts on Economy and Society

In view of the fact that national health indicators can reflect the overall development level and people's quality of life of a country to a certain extent, the literature review should also be extended to the broader research topic of the impact of ICTs on the economy and society.

Cisco conducted a time-series analysis to explain the positive impact of ICT investment on UK economic growth (1999–2000). It has been found that the positive impact of ICT investment is particularly evident in the job market and is achieved through human capital restructuring. Likewise, Chu [41] found that from 1987 to 2001, the profit generated by New Zealand's IT service industry was positively correlated with GDP growth. By employing Toda–Yamamoto Granger causality approach, Solarin et al. [42] investigated the impact of ICTs, financial development and economic growth on electricity consumption in Malaysia and found a positive feedback effect between ICTs and electricity consumption. Meanwhile, in the trade research area, ICTs, as the carrier of digital trade, also have been proved to be able to promote green total factor productivity (GTFP) combined with human capital factor and R&D factor [43].

In order to make comparative studies on the national ICT level of different countries, Northrop [44] introduced a path model to examine the association among economic factors, social infrastructure and information infrastructure. The model used multiple regression analysis and path analysis to study the factors influencing the transnational differences in computer penetration.

Multiple similar papers have mentioned how an economy can benefit from the development of ICTs. First of all, NIA [45] proposed the positive impact of ICTs on national competitiveness by studying how the status of cross-national ICTs is related to the national competitiveness indicators of the World Economic Forum. Secondly, in a study of 19 countries, OECD (2008) indicated that the popularity of broadband technology was related to GDP growth. Finally, it threw light on the importance of public investment based on the analysis of the broadband technology opportunity program.

Apart from their economic role, ICTs also exert a profound influence on various social aspects. Park and Lee [46] discovered specific linkages between different forms of social capital and different forms of ICTs, suggesting a positive role of cell phone use for interpersonal purposes in facilitating bonding social capital, and that of computer use for political and information purposes in promoting bridging social capital. According to Synowiec [47], ICTs contribute to rural development by creating sources of income and granting access to education. Edinyang et al. [48] believed that in the days of information explosion, social development in Nigeria can be enhanced by ICTs as a strong catalyzer for knowledge integration. In addition, the dissemination of ICTs sees its own part in innovating social protection schemes [49], bolstering family solidarity [50], and developing home-based business communities [51].

### 2.4. Summary of the Literature

In view of this background, we can conclude that the positive link between ICTs and public health outcomes has been widely discussed. However, most existing studies generally focus on case studies and the introduction of specific technologies in individual countries or even in a specific location within a country. In the research of related fields, some focus on the correlations among variables such as ICTs, e-Health (and related policies), digital divide, public health expenditure and a number of health indicators, and some conduct cluster analysis of countries in specific regions based on these indicators [52]. Although these studies provide detailed and rich data representation, their analysis level does not rise to the level of broader samples. Moreover, previous researchers have not studied whether ICTs indirectly affect health indicators by influencing the economy and society. After all, e-Health mentioned above is actually one of the social impacts of ICTs.

Based on prior studies, this research further subdivides ICT factors to refine the granularity of variables. Grounded on the four dimensions of NRI released by World Economic Forum, ICT environment, ICT readiness, and ICT usage three dimensions are selected as independent variables. Four health indicators from the World Bank database are selected as dependent variables. This research selects ICT economic impact and ICT social impact from the NRI as two mediating variables to represent the fourth NRI dimension, ICT impact, which is the first indicator adopted in all similar studies. It is also the first time that they have been used as mediating variables to explore their role in the relationships between ICT indicators and health levels via the mediated effect model.

## 3. Research Model and Research Hypothesis

### 3.1. ICT Factors and National Health Outcomes

All the ICT factors used in this study are extracted from the NRI from the Global Information Technology Report, which has been annually released for the last decade. The World Economic Forum, in collaboration with INSEAD, initially began this project to explore the impact of ICTs on productivity and development, as a component of the Forum's research on competitiveness. To this end, over the past decade, the NRI has been measuring the degree to which economies across the world leverage ICTs for enhanced competitiveness. During this period, it has been helping policymakers and relevant stakeholders to track their economies' strengths and weaknesses as well as their progress over time. It is also a solid and substantial data source for the academic community to conduct empirical research.

NRI is a comprehensive index composed of 4 subindices, 10 pillars, and 53 independent indicators distributed on different pillars. The main data providers are the International Telecommunication Union (ITU), UNESCO, and other UN agencies, as well as the World Bank. The other half comes from the executive opinion survey of the World Economic Forum.

The four subindices of NRI are ICT environment, ICT readiness, ICT usage, and ICT impact. In this study, three subindices, ICT environment, ICT readiness, and ICT usage, are selected as the independent variables. The ICT environment subindex gauges the friendliness of a country's market and regulatory frameworks and their ability to support high levels of ICT uptake and the development of entrepreneurship; it also gauges the presence of innovation-prone conditions needed to maximize the potential impacts of ICTs in boosting the economy's competitiveness and its citizens' well-being. The ICT readiness subindex measures the degree to which a society is prepared to make good use of an affordable ICT infrastructure and digital content. The ICT usage subindex assesses the individual efforts of the main social agents—that is, individuals, business, and governments—to increase their capacity to use ICTs, as well as their actual use in their day-to-day activities with other agents.

The dependent variables selected in this research, health indicators, are from MDGs and World Development Indicators. These indicators are the under-five mortality rate, maternal mortality ratio, adolescent fertility rate, and life expectancy at birth. They are widely recognized and applied by international organizations such as the United Nations, and have also been used many times in previous studies.

#### 3.1.1. Under-Five Mortality Rate

Many studies have highlighted the role of ICTs in supporting the delivery of health services, especially in maternal and child health. In terms of Goal 4-reduce child mortality from MDGs, one of the main reasons is the lack of knowledge about childhood diseases, which applies to both developed and developing countries. Access to information through the Internet, mobile communications, radio, and other ICT applications can help parents and doctors find ways to treat sick children better. In developed countries like the United States, a telemedicine program for parents of infants reports that they have 10% higher quality of care than those who do not use telemedicine systems. In developing countries, there is already global public health information and education based on SMS. Studies have shown that the percentage of parents using ICT-based health tools can measure the impact of ICTs on improving the health of infants and children, thereby reducing their mortality. Specifically, in terms of ICT environment, the friendlier a country's market and regulatory framework is, or the better its ability to support high levels of ICT uptake and entrepreneurial development is, the greater the support of ICTs for medical and health services will be, making it possible for parents and doctors, as well as hospitals, to take more effective measures to reduce child mortality. Similarly, if a country is well prepared to leverage affordable ICT infrastructure and digital content, or it has made significant efforts to improve its ability to use ICTs, it will be able to integrate ICTs with healthcare services better, which will lead to better child mortality reduction at the country-wide level. Therefore, we can make the following hypotheses:

1. H1 : ICT factors are negatively related with under-five mortality rate.
2. H1a : ICT environment is negatively related with under-five mortality rate.
3. H1b : ICT readiness is negatively related with under-five mortality rate.
4. H1c : ICT usage is negatively related with under-five mortality rate.

#### 3.1.2. Maternal Mortality Ratio

In terms of Goal 5-improve maternal health from MDGs, 99% of maternal deaths occur in developing countries. In India, SISU Samrakshak (SSK) refers to a child protector jointly developed by the United Nations Children's Fund (UNICEF) Hyderabad Field Office, CoOptions Technologies Ltd. And the AP government in 2000. SSK deploys ICTs in regional languages to impart health, hygiene, and sanitation knowledge to illiterate communities through audio, pictures, videos, touch screens, and culturally appropriate images. It provides basic information on the different stages of a child from pregnancy to adolescence, women's health during pregnancy, nutrition, child development, safe motherhood, immunization, common diseases, and their remedies. It treats mothers as primary caregivers but allows key actors (such as front-line government workers in the health, nutrition, and education sectors) to promote community learning. Maternal mortality is a key factor in measuring the overall health of a country. If a country has the ability to support higher levels of ICT uptake and the development of entrepreneurship, the country's ICT hardware facilities and related application level will be higher, and ICTs will provide more support for social medical and health services, so that women themselves, families, doctors, and hospitals are likely to take more effective measures to reduce maternal mortality. Likewise, the full preparation to make good use of the affordable ICT infrastructure and digital content, and the higher capacity to use ICTs, will enable the whole society to better reduce maternal mortality, given that the dissemination and use of information, knowledge, and measures on maternal care will be more effective. Therefore, we can make the following hypotheses:

1. H2 : ICT factors are negatively related with maternal mortality ratio.
2. H2a : ICT environment is negatively related with maternal mortality ratio.
3. H2b : ICT readiness is negatively related with maternal mortality ratio.
4. H2c : ICT usage is negatively related with maternal mortality ratio.

#### 3.1.3. Adolescent Fertility Rate

The adolescent fertility rate is mainly used to reflect the education level of adolescents, including basic education and sex education. The high adolescent birth rate means fewer adolescents are in education. In addition, early childbearing itself is associated with complications and less access to post-natal health care. Globally, the adolescent birth rate among women aged 15–19 has fallen 21% since 2000. However, two-thirds of all countries still have high adolescent birth rates. In general, the spread and application of ICTs can assist in the provision of health information through online health services, and then help the adolescent population to continue their education at a higher level, take preventive measures, thus reduce fertility rates. If the country offers friendly market and regulatory frameworks, and encourages business innovation and practice, it can create a good environment to improve the number of years and levels of education of young people. Meanwhile, the better readiness and preparation of ICTs, or the wider and deeper use of ICTs, will enable the whole society to better reduce the adolescent fertility rate, given that this will help popularize basic education and sex education for young people. Therefore, we can make the following hypotheses:

1. H3 : ICT factors are negatively related to adolescent fertility rate.
2. H3a : ICT environment is negatively related to adolescent fertility rate.
3. H3b : ICT readiness is negatively related to adolescent fertility rate.
4. H3c : ICT usage is negatively related to adolescent fertility rate.

#### 3.1.4. Life Expectancy at Birth

Life expectancy at birth (or life expectancy for short) is an important indicator of life. A key goal of improving the national health is to increase people's life expectancy, and the use of ICTs can make a huge difference here. On one hand, ICT devices and applications can provide health workers with ICT-assisted functions to collect, record, and share information about health conditions of patients, thereby effectively assisting medical and treatment decision-making, improving medical standards, and resultingly increasing care rates. And on the other, ICTs can contribute overall to this goal by providing health-related information to the public through, for example, online health, and through follow-up activities to educate the public. If a country has an advanced and mature ICT environment, then it has a higher level of ICT hardware facilities and related applications, ICT support for social medical and health services will also be greater. As a result, the general population can generally benefit from this and thus increase life expectancy. Likewise, the higher readiness of ICTs, or the wider and deeper use of ICTs, will enable the whole society to better improve life expectancy, given that the dissemination and use of information, knowledge and measures on healthcare will be more effective. Therefore, we can make the following hypotheses:

1. H4 : ICT factors are positively related to life expectancy at birth.
2. H4a : ICT environment is positively related to life expectancy at birth.
3. H4b : ICT readiness is positively related to life expectancy at birth.
4. H4c : ICT usage is positively related to life expectancy at birth.

### 3.2. ICT Impact and the Mediation Role

ICT factors can directly improve the national health levels, but at the same time, we need to note that ICT factors are playing a different role in improving the national health levels with the direct role of treatments or medicines. They are playing a role in making the health information processing more efficient and effective, making the treatment process more convenient and intelligent, improving the economy of the nation, improving the well-being of society, and thus indirectly enhancing the national health levels. Therefore, we can hypothesize that ICT factors have different mechanisms of action, both direct and mediated, for the improvement of national health status.

In this study, we use ICT impact from NRI as mediating variable to characterize the mediating mechanism between ICT factors and national health levels. We divide this mediating mechanism into two aspects, ICT economic impact and ICT social impact, to measure the extensive economic and social impact of ICT to enhance competitiveness and welfare, reflecting the transition to ICT and technology-sensitive economy and society.

Economic impact measures the impact of ICTs on competitiveness, which is due to technological and non-technological innovation in the form of patents, new products or processes, and organizational practices. It also measures the overall shift of an economy towards knowledge-intensive activities.

Social impact aims to assess the improvement in well-being due to the impact of ICTs on the environment, education, energy consumption, health progress, or more active citizen participation. At present, due to limited data, this pillar focuses on measuring the extent to which governments have improved the use efficiency of ICTs and provided more and more online services to their citizens, thereby facilitating their online participation. It also assesses the extent of ICT application in education, reflecting the potential benefits of ICT use in education.

As mentioned above, ICTs can influence a country's economy and society and thus its overall level of development, including economic growth and the job market, sources of income and educational opportunities [47], and, of course, the level of national health that we focus on here. Therefore, we can formulate the following hypothesis:

H5 : ICT impact has a mediated effect between ICT factors and national health outcomes.

In this study, there are three independent variables, two intermediary variables, and four dependent variables. Due to the large number of variables and limited space, all sub-hypotheses of H5 are not listed here.

### 3.3. Theoretical Model

Totally, the purpose of this cross-national study is to empirically evaluate the two related research questions: Do ICT factors influence national health outcomes of a country over time? Do economic and social impacts of ICTs mediate the relationship between ICT factors and national health outcomes?

In addition, considering that national income will greatly affect national health, we refer to the previous literature and add GDP by country (from the World Bank) into our model as a control variable.

Based on the above discussion, this research establishes a research model, as shown in Figure 1:

## 4. Empirical Research

### 4.1. Variables and Data Measurement

This research collect data from World Bank and World Economic Forum Global Information Technology Report from 2012 to 2016. To obtain a set of balanced panel data, we took the intersection of the two databases and finally obtained 141 countries as the study samples (see Table1 for the list of countries). These 141 countries represent different continents and different economic levels and are generally representative. Regarding the measurement of the three independent variables, based on the preceding literature and analysis, this paper measures ICT environment using the pillar business and innovation environment from NRI, measures ICT readiness using the pillar affordability from NRI, and measures ICT usage using the pillar individual usage from NRI.

In order to obtain effective results in subsequent data analysis, the dependent variables and the control variable GDP are reported in logarithmic form due to the large differences among sample countries and scattered sample data. All the variables are organized in Table 2.

### 4.2. Mediated Effect Model

The mediated effect model originates from the research in the field of psychology. Considering the influence of independent variable *X* on the dependent variable *y*, if *X* influences *Y* by influencing variable *M*, then *M* is called the mediating variable. The following regression equations and the model shown in Figure 2 can be used to describe the relationship between variables

(1) $$\begin{array}{c} \;Y=i+cX+e_{1}, \end{array}$$

(2) $$\begin{array}{c} M=i+aX+e_{2}, \end{array}$$

(3) $$\begin{array}{c} Y=i+c^{'}X+bM+e_{3}. \end{array}$$

Coefficient *c* of equation (1) is the total effect of independent variable *X* on the dependent variable *Y*. Coefficient *a* of equation (2) is the effect of independent variable *X* on mediating variable *M*. Coefficient *b* of equation (3) is the effect of mediating variable *M* on the dependent variable *Y* after controlling the influence of independent variable *X*. Coefficient *c'* is the direct effect of independent variable *X* on dependent variable *Y* after controlling the influence of intermediate variable *m*. *e*_*1*_, *e*_*2*_, and *e*_*3*_ are residuals.

The most commonly used method to test the mediated effect is causal step regression [53, 54]:

- Test coefficient *c* of equation (1). If coefficient *c* is not significant, then there is no need for the mediation test.
- Test coefficient *a* of equation (2) and coefficient *b* of equation (3), which is called the joint significance test [55]. If coefficient *c* is significant as well as coefficients *a* and *b*, then the mediated effect is significant, and proceed to step iii. If *a* or *b* or both are not significant, the Sobel test is performed to further determine whether there is a mediated effect.
- Test coefficient *c'* of equation (3). If *c'* is significant, the mediated effect is partial; otherwise, it is complete.

The mediated effect model is used as the main mechanism in this paper, in which three ICT factor variables are independent variables (X), two ICT impact variables are mediating variables (M), and four national health outcome variables are dependent variables (Y). At the same time, the balanced panel data of 141 countries from 2012 to 2016 are used in this paper, so the mediation test of panel data will be performed.

### 4.3. Data Analysis

The panel data analysis and corresponding mediated effect analysis are conducted in STATA. Considering individual differences between different countries, this study adopts fixed effect model to verify panel data. All the results are shown in Tables 3–6.

For the first step, the associations between ICT factors and national health outcomes are tested. The association between the ICT factors and the four health indicators is summarized in Table 3.

The results show that ICT environment has a significant negative impact on under-five mortality rate, maternal mortality ratio, and adolescent fertility rate. H1a, H2a, and H3a are confirmed, but H4a is not. The impact of ICT readiness on four national health indicators is not confirmed. ICT usage has a significant impact on the four health outcome indicators, meaning that H1c, H2c, H3c, and H4c are confirmed. Meanwhile, the influence of improving national GDP on the above four health outcome indicators is also confirmed.

Therefore, it can be proved that ICT factors have a significant role in promoting the overall national health. Improving ICT environment and ICT usage can effectively reduce under-five mortality rate, maternal mortality ratio, and adolescent fertility rate, while improving ICT usage can promote life expectancy at birth.

The hypotheses that are not confirmed in the first step will not proceed to subsequent mediation tests, and we can directly affirm that there is no mediated effect regarding these hypotheses. Therefore, the following tests will explore whether the two mediating variables, ICT economic impact and ICT social impact, have mediated effects on the relationship between ICT environment and under-five mortality rate, maternal mortality ratio, and adolescent fertility rate, and whether they can mediate between the independent variable ICT usage and the four dependent variables.

The second step is the mediation test, which should test the coefficient a in the model equation (2).  Table 4 shows the relationship between ICT factors and the economic and social impact of ICTs.

It can be seen that the correlation between ICT environment and ICT economic impact, the correlation between ICT environment and ICT social impact, and the correlation between ICT usage and ICT social impact are all positively significant, that is, the coefficient “a” is significant, which can enter step 3 of the mediation test.

However, the correlations between ICT usage and ICT economic impact are not significant, so the Sobel test will be performed to further explore the possible mediated effect.

After step 2, we enter the third step of mediation test, which is to test the coefficient *b* and the coefficient c' in the model formula (3).  Table 5 and Table 6 show the results.

Tables 5 and 6 show that when independent variables are controlled, the ICT economic impact has no significant effect on the four health indicators, meaning that their coefficient *b* is not significant. Therefore, all the mediated effects with ICT economic impact as the mediating variable will enter the subsequent Sobel test.

Meanwhile, we can see that when under-five mortality rate and adolescent fertility rate are dependent variables, and independent variables ICT environment and ICT usage and mediating variable ICT social impact are entered the regression model, their coefficients *b* and c' are all significant. Therefore, it can be directly determined that for dependent variables under-five mortality rate and adolescent fertility rate, ICT social impact has a partial mediated effect on their relationship with ICT environment and ICT usage. However, for the dependent variables maternal mortality ratio and life expectancy at birth, it is still unclear whether ICT social impact has a mediated effect, so further Sobel test is needed.

Now, we conduct a Sobel test on the above hypotheses where the mediated effect may exist but so far cannot be confirmed. During the Sobel test, we still follow the fixed effect test rule of panel data and add dummy variables representing the national individual effect into the regression model as control variables. The test results show that only ICT economic impact has a mediated effect between ICT environment and under-five mortality rate (Sobel *p* value = 0.377, Goodman-1(Aroian) *p* value = 0.0407, Goodman-2 *p* value = 0.0348). However, the proportion of total effect that is mediated is minus, indicating that the suppression effect occurs and the mediated effect cannot be confirmed.

In a nutshell, the partial mediated effect that has been confirmed in previous analyses is reconfirmed in the Sobel test. The proportion of the partial mediated effect and key information is summarized as follows:

The final results of the mediated effect model are displayed in Table 7, indicating that part of H5 is proved. First, all evident mediated effects are partial mediation. This is not hard to understand. Previous research has suggested that complete mediation is rare [56]. When we conclude a complete mediation, we actually rule out exploring other mediated effects in the future [57]. Preacher and Hayes [58] called for the abandonment of the concept of complete mediation and regarded all mediated effects as partial mediation. The results of our study further verify this point.

Second, the results show that ICT environment and ICT usage can influence both under-five mortality rate and adolescent fertility rate via ICT social impact. In other words, ICT environment and ICT usage can reduce under-five mortality rate and adolescent fertility rate by improving the social impact of ICTs. Although it can be seen from Table 6 that the proportion of total effect that is mediated is not high, indicating the effects of the independent variables on the dependent variables are the results of a combination of multiple factors, and the ICT social impact plays a relatively weak mediating role here. At the same time, the mediated effect of ICT social impact on maternal mortality ratio and life expectancy at birth is not confirmed. The mediated effect of ICT economic impact is not confirmed either.

Based on the above studies, all the results of hypothesis testing are summarized in Table 8:

## 5. Discussion

### 5.1. ICTs and National Health Outcomes

This paper is highly relevant to the studies of the relationship between ICT and health outcomes, especially the cross-national research methods and conclusions, which are the most crucial to enlightening this research. The unit of analysis is a national-level characteristic. Thus, the outcome of this research should be applied to the explanation of national development, not individual, within a particular country to avoid ecological fallacy.

Our results indicate that overall ICT factors substantially facilitate national public health delivery. ICT factors are usually discussed as a whole and as one independent variable in the previous literature, mostly proved conducive to promoting health outcomes. This paper, however, divides ICT factors into three detailed dimensions of ICT environment, ICT readiness, and ICT usage based on NRI and finds that not all ICT factors have a significant impact.

ICT environment shows a significant role in promoting national health outcomes, especially in reducing under-five mortality rate, maternal mortality ratio, and adolescent fertility rate. This indicates that a country can effectively promote the development of ICT infrastructure and related applications by encouraging and supporting innovation, entrepreneurship and business, which leads to greater assistance and support of ICTs for social medical and health services, bringing more widespread benefits to the population and thus effectively reducing under-five mortality rate, maternal mortality ratio, and adolescent fertility rate. Exception occurs in that ICT environment has no significant impact on life expectancy at birth. A possible reason is that what ICT environment determines is the level of maturity and advancement of a country's market and business environment, which to some extent influences the national economic development, but may make little direct impact on life expectancy at birth. Another possible reason is that the conclusions of this study are based on data from 2012 to 2016, and due to the specificity of the data from this time period, it is not yet possible to effectively prove that ICT environment has a positive effect on the life expectancy at birth of the population, so the verification of this hypothesis needs to be confirmed by data from other subsequent years.

ICT readiness measures the degree to which a society is prepared to make good use of ICT infrastructure and related applications. The empirical results of this study suggest that its impact on improving national health is only marginal and statistically insignificant. One possible reason is that ICT readiness is different from ICT usage; it simply indicates the readiness of the country and society for future ICT use, but is distinct from the direct contribution that ICT usage can bring to national health levels. Therefore, the true impact of ICT readiness on national health outcomes needs further testing.

ICT usage measures the penetration and dissemination of ICTs, including the use of hardware facilities, software applications, and data. Comparatively speaking, the use of ICTs by individuals has the most direct and effective effect on the improvement of individual health outcomes. Therefore, ICT usage has the most significant impact on reducing under-five mortality rate, maternal mortality ratio and adolescent fertility rate, as well as promoting life expectancy at birth.

In general, ICTs are playing a significant role in improving national health, especially in developing countries. When ICTs are combined with healthcare, they can make a key contribution to improve the lives and well-being of people around the world. They can also support improvements in health development. With the rapid development of ICTs and online health, relevant successful cases abound in many less developed regions of the world.

### 5.2. Mediated Effects

ICTs are not medicines, vaccines, or health policies, rather ICTs are technologies that enable the processing of health information much more efficiently and effectively. However, ICT factors have different acting mechanisms on health outcomes. Some ICT factors use economic influence as a mediator, some use social influence, and some may directly influence health outcomes or may use other mediating variables not included in this paper.

In terms of the empirical results of the mediated effect, the cross-comparison of the two mediating variables shows that while ICT economic impact only exerts its influence in the economic field, ICT social impact can have an effect in a broader field of people's daily life. Relevant indicators are access to basic ICT services, Internet access in schools, ICT use and government effectiveness, and people's online engagement index. ICT infrastructure first permeates through the social life of a country, and then, as the country's social life thrives, the health of its people gradually improves. This makes the influence and mediated effect of ICT social impact on national health outcomes more significant.

When ICT social impact is used as the mediating variable, ICT environment and ICT usage were the two factors with the most significant results. Both ICT environment and ICT usage can reduce under-five mortality rate and adolescent fertility rate by improving ICT social impact. That is, by improving and optimizing the country's friendliness of a country's market and regulatory frameworks, and by further popularizing usage of ICTs, it is possible to bring improvements in the well-being of the environment, education, energy consumption, or more active civic participation as a result of the use of ICTs. Thus, we can conclude that a possible path is that ICT infrastructure lays a solid foundation for the widespread dissemination of social services, including neonatal care education, government support for childbirth, and abundant Internet resources, and thus effectively improves national health outcomes. This is mainly reflected in lowering under-five mortality rate and adolescent fertility rate.

However, the mediated effect of ICT usage on maternal mortality ratio and life expectancy at birth through ICT social impact is not confirmed. Although empirical results show that ICT usage does have a direct impact on maternal mortality ratio and life expectancy at birth, there is not enough evidence to prove that this impact can have an indirect effect through ICT social impact. One possible reason is that ICT social impact is too limited to cover the major factors influencing maternal mortality ratio and life expectancy at birth. Under the NRI, ICT social impact is measured by four indicators confined to ICTs' contributions to the accessibility of basic services, Internet use for learning purposes in school, quality of government services, and the public E-participation. Maternal mortality ratio, however, is much affected by socioeconomic disparity, urban-rural differences, women empowerment, and equity, as well as social norms and culture [59, 60], which are hardly encompassed by the NRI. Likewise, ICT social impact under the NRI overlaps little with the broad determinants of life expectancy at birth, including economy, literacy, nutritional status, and political regime [61]. Thus, limitations in the measurement of the variable ICT social impact are a possible reason for the failure of this study to effectively confirm its mediating effect between ICT use and maternal mortality ratio and life expectancy at birth.

Meanwhile, the mediated effect of ICT environment on maternal mortality ratio through ICT social impact is not confirmed. Although empirical results show that ICT environment does have a direct impact on maternal mortality ratio. One possible reason for this, in addition to the fact that the social impact of ICTs, as mentioned above, is too limited to cover the main factors influencing maternal mortality ratio, is that ICT environment, the indicator of a country's business and market environment, which gauges the normative nature of regulatory framework and the presence of innovation-prone conditions, may channel its influence primarily through corporate, market, or even political factors rather than ICT social impact.

Finally, as mentioned above, unlike that of ICT social impact, the mediated effect of ICT economic impact is not confirmed. One possible reason is that according to the data source of this study, ICT economic impact is measured by ICT impact on business model, ICT patent application, ICT impact on organizational model, and the number of knowledge-intensive jobs. It is easy to see that ICT economic impact is mainly confined to the business sector. The important impacts of ICTs are multidimensional, and while previous empirical tests show that they do affect national health outcomes, many of these impacts are not currently being translated into or reflected in business. As a result, the mediated effect of ICT economic impact in this process becomes difficult to define and measure. Although not in line with our hypotheses, we can accept that the mediated effect is relatively weak in our research paradigm. Still, we hold the possibility that the measurements of those variables can be insufficient or inappropriate and leave space for future studies.

In general, measuring the impact of ICTs is a complex task, and the development of rigorous quantitative data for this purpose is still in its infancy. It is difficult to precisely define the impact, which is one of the main obstacles, because ICTs have proved transformative in many aspects of the economy and society, affecting not only the results but also the process of providing products and services. Therefore, it is difficult and expensive to develop indicators to measure these dimensions, especially when a large number of emerging countries are involved. Moreover, even if the area of impact can be identified, it is not necessarily easy to trace a particular impact back to all its original sources. The often observed economic and social impacts are the result of a tight network of interacting factors, and ICT is only one of them. As a result, many aspects of ICT impact (such as health environment) cannot be covered, especially when these impacts are not translated into commercial activities. Therefore, the ICT impact index should be regarded as an ongoing work. With the emergence of all kinds of new data, it will continue to develop and improve new dimensions.

## 6. Conclusion, Limitation, and Future Research

Based on the above studies, this research clarifies that ICT factors can influence national health outcomes of a country over time and ICT social impact can play an important partial mediating role between them.

The contributions of this study can be categorized into theoretical and practical ones. Theoretically, previous studies on ICTs and health development are mostly conceptual, or remain at the micro-level, focusing on the actual operation of technology. This study raises the theoretical altitude to a micro-level, introducing a wider sample of countries from the United Nations when a large number of fellow studies only look at EU, other regional organizations or even just individual countries. Second, on top of ICT factors, we bring in ICT impacts as mediations in our model, which is an innovation in the area. We hope it can serve as a good beginning for researchers to try other theoretical models and make them more sufficient and accurate. Finally, the study aims to review the realization of MDGs (2000–2015) and provide inspiration for SDGs (2015–2030). SDGs have 17 new development goals and will continue to guide the global development work in 2015–2030 after the expiration of the 2000–2015 MDGs. The goal of sustainable development is to solve the development problems of society, economy, and environment in a comprehensive way from 2015 to 2030 and turn to the road of sustainable development. Our study can lay the foundation for future research on SDGs, as well as for the comparative study of MDGs and SDGs.

Practically, this study aims to help global policymakers formulate health resource allocation and investment strategies, especially in the fields of healthcare and technology in developing countries. As we provide a new perspective to see how ICT factors associate with its impact, developing countries can use it as a guide to get financial assistance from or cooperate with other countries or organizations to improve health deliveries from their weakest areas with the most urgent needs according to their own conditions. To promote the implementation of SDGs in the next stage, we suggest integrating and determining priorities in national development and health promotion programs and strategies, adjusting policies for basic infrastructure deployment, facilitating donor coordination and cooperation mechanisms, strengthening the participation of the private sector, and coordinating resource mobilization mechanisms.

This study has the following limitations. First of all, this study uses the secondary data research method. The data is sourced from the annual macro data released by authoritative international government organizations which always need a long cycle to collect and the completeness is not enough. Due to the redesign of the NRI system, the complete data available are only from 2012 to 2016. The NRI was suspended during 2017 and 2018 for a redesign. Data from 2019 onwards comes from a new NRI system, which is incompatible with the previous ones. Therefore, 141 countries from 2012 to 2016 are selected as samples. The total observation values of each group regression range from 660 to 662. The sample size is comparatively small. In the future, with the development of innovative technologies and the completeness of data collected by various international government organizations, ongoing tracking and research could be considered, starting with data from 2019. A before-and-after study could also be considered to further explore the ongoing changes in national health levels as ICT use and penetration increase.

Secondly, the mediated effect model in this study aims to explore the role of the economic impact and social impact of ICTs on the relationship between ICTs and national health outcomes. However, this model is still in its original stage and further correction and adjustment are needed. In addition to the mediated effect, the moderating effects should be explored, and variable selection and data sources can be constantly updated in the future.

## Figures and Tables

**Figure 1:** Research model.

**Figure 2:** Mediated effect model (Baron and Kenny, 1986).

**Table 1:** The list of countries.

1	Albania
2	Algeria
3	Angola
4	Argentina
5	Armenia
6	Australia
7	Austria
8	Azerbaijan
9	Bahrain
10	Bangladesh
11	Barbados
12	Belgium
13	Belize
14	Benin
15	Bhutan
16	Bolivia
17	Bosnia and Herzegovina
18	Botswana
19	Brazil
20	Brunei Darussalam
21	Bulgaria
22	Burkina Faso
23	Burundi
24	Cambodia
25	Cameroon
26	Canada
27	Chad
28	Chile
29	China
30	Colombia
31	Costa Rica
32	Croatia
33	Cyprus
34	Czech Republic
35	Denmark
36	Dominican Republic
37	Ecuador
38	El Salvador
39	Estonia
40	Ethiopia
41	Finland
42	France
43	Gabon
44	Gambia
45	Georgia
46	Germany
47	Ghana
48	Greece
49	Guatemala
50	Guinea
51	Guyana
52	Haiti
53	Honduras
54	Hungary
55	Iceland
56	India
57	Indonesia
58	Iran, Islamic Rep.
59	Ireland
60	Israel
61	Italy
62	Jamaica
63	Japan
64	Jordan
65	Kazakhstan
66	Kenya
67	Korea, Rep.
68	Kuwait
69	Kyrgyz Republic
70	Lao PDR
71	Latvia
72	Lebanon
73	Lesotho
74	Liberia
75	Libya
76	Lithuania
77	Luxembourg
78	Madagascar
79	Malawi
80	Malaysia
81	Mali
82	Malta
83	Mauritania
84	Mauritius
85	Mexico
86	Moldova
87	Mongolia
88	Montenegro
89	Morocco
90	Mozambique
91	Myanmar
92	Namibia
93	Nepal
94	Netherlands
95	New Zealand
96	Nicaragua
97	Nigeria
98	Norway
99	Oman
100	Pakistan
101	Panama
102	Paraguay
103	Peru
104	Philippines
105	Poland
106	Portugal
107	Puerto Rico
108	Qatar
109	Romania
110	Russian Federation
111	Rwanda
112	Saudi Arabia
113	Senegal
114	Serbia
115	Seychelles
116	Sierra Leone
117	Singapore
118	Slovak Republic
119	Slovenia
120	South Africa
121	Spain
122	Sri Lanka
123	Suriname
124	Sweden
125	Switzerland
126	Tajikistan
127	Tanzania
128	Thailand
129	Timor-Leste
130	Trinidad and Tobago
131	Tunisia
132	Turkey
133	Uganda
134	Ukraine
135	United Arab Emirates
136	United Kingdom
137	United States
138	Uruguay
139	Vietnam
140	Zambia
141	Zimbabwe

**Table 2:** Data sources and descriptive analysis.

Category	Variable	Content	Data source	Method	*N*	Mean	Sd	Min	Max
Dependent variables	Under-five mortality rate	Under-five mortality rate/MDGs-goal 4	World bank	Ln	700	2.76	1.13	0.79	4.99
	Maternal mortality ratio	Maternal mortality ratio/MDGs-goal 5	World bank	Ln	700	2.54	1.07	0.59	4.61
	Adolescent fertility rate	Adolescent fertility rate/MDGs-goal 5	World bank	Ln	705	3.38	1.07	0.38	5.19
	Life expectancy at birth	Life expectancy at birth/World development indicators	World bank	Ln	705	4.28	0.12	3.86	4.43

Independent variables	ICT environment	NRI pillar: business and innovation environment	WEF—the global information technology report	n/a	671	4.24	0.69	2.36	5.97
	ICT readiness	NRI pillar: affordability	WEF—the global information technology report	n/a	662	4.9	1.32	1	7
	ICT usage	NRI pillar: individual usage	WEF—the global information technology report	n/a	671	3.77	1.55	1.3	6.86

Mediating variables	ICT economic impact	ICT impact-economic impact	WEF—the global information technology report	n/a	671	3.45	0.95	1.83	6.15
	ICT social impact	ICT impact-social impact	WEF—the global information technology report	n/a	671	3.96	1.01	1.7	6.28

Control variables	GDP	GDP (constant 2010 US$)	World bank	Ln	705	24.91	1.99	20.89	30.55

**Table 3:** Associations between ICT factors and national health outcomes.

Variables	(1)	(2)	(3)	(4)
	Under-five mortality rate	Maternal mortality ratio	Adolescent fertility rate	Life expectancy at birth
ICT environment	−0.0575^*∗∗∗*^	−0.0547^*∗∗∗*^	−0.0680^*∗∗∗*^	0.00243
	(0.0134)	(0.0128)	(0.0168)	(0.00256)
ICT readiness	−0.00257	−0.00312	0.00680^*∗∗*^	0.000210
	(0.00258)	(0.00246)	(0.00325)	(0.000493)
ICT usage	−0.0661^*∗∗∗*^	−0.0708^*∗∗∗*^	−0.0555^*∗∗∗*^	0.00406^*∗∗∗*^
	(0.00639)	(0.00611)	(0.00804)	(0.00122)
GDP	−0.425^*∗∗∗*^	−0.346^*∗∗∗*^	−0.234^*∗∗∗*^	0.0850^*∗∗∗*^
	(0.0342)	(0.0327)	(0.0431)	(0.00654)
Constant	13.84^*∗∗∗*^	11.67^*∗∗∗*^	9.667^*∗∗∗*^	2.130^*∗∗∗*^
	(0.835)	(0.798)	(1.051)	(0.160)
Observations	660	660	662	662
R-squared	0.626	0.618	0.364	0.438
Number of id	140	140	141	141

Standard errors in parentheses ^*∗∗∗*^*p* < 0.01, ^*∗∗*^*p* < 0.05, ^*∗*^*p* < 0.1

**Table 4:** Associations between ICT factors and ICT Impacts.

Variables	(5)	(6)
	ICT economic impact	ICT social impact
ICT environment	0.257^*∗∗∗*^	0.373^*∗∗∗*^
	(0.0497)	(0.0772)
ICT usage	0.00795	0.233^*∗∗∗*^
	(0.0237)	(0.0369)
GDP	0.00485	0.852^*∗∗∗*^
	(0.127)	(0.197)
Constant	2.176	−19.79^*∗∗∗*^
	(3.105)	(4.817)
Observations	662	662
R-squared	0.074	0.334
Number of id	141	141

Standard errors in parentheses ^*∗∗∗*^*p* < 0.01, ^*∗∗*^*p* < 0.05, ^*∗*^*p* < 0.1

**Table 5:** Mediated effect model (MV is the ICT economic impact).

Variables	(7)	(8)	(9)	(10)
	Under-five mortality rate	Maternal mortality ratio	Adolescent fertility rate	Life expectancy at birth
ICT environment	−0.0644^*∗∗∗*^	−0.0592^*∗∗∗*^	−0.0725^*∗∗∗*^	
	(0.0137)	(0.0131)	(0.0173)	
ICT usage	−0.0665^*∗∗∗*^	−0.0711^*∗∗∗*^	−0.0556^*∗∗∗*^	0.00411^*∗∗∗*^
	(0.00637)	(0.00610)	(0.00804)	(0.00121)
ICT economic impact	0.0270^*∗∗*^	0.0175	0.0172	-0.00651^*∗∗∗*^
	(0.0119)	(0.0114)	(0.0149)	(0.00224)
GDP	−0.424^*∗∗∗*^	−0.346^*∗∗∗*^	−0.234^*∗∗∗*^	0.0850^*∗∗∗*^
	(0.0341)	(0.0327)	(0.0431)	(0.00649)
Constant	13.76^*∗∗∗*^	11.62^*∗∗∗*^	9.630^*∗∗∗*^	2.145^*∗∗∗*^
	(0.832)	(0.798)	(1.051)	(0.159)
Observations	660	660	662	662
R-squared	0.630	0.619	0.365	0.447
Number of id	140	140	141	141

Standard errors in parentheses ^*∗∗∗*^*p* < 0.01, ^*∗∗*^*p* < 0.05, ^*∗*^*p* < 0.1

**Table 6:** Mediated effect model (MV is the ICT social impact).

Variables	(11)	(12)	(13)	(14)
	Under-five mortality rate	Maternal mortality ratio	Adolescent fertility rate	Life expectancy at birth
ICT environment	−0.0520^*∗∗∗*^	−0.0504^*∗∗∗*^	−0.0617^*∗∗∗*^	
	(0.0136)	(0.0130)	(0.0172)	
ICT usage	−0.0627^*∗∗∗*^	−0.0681^*∗∗∗*^	−0.0515^*∗∗∗*^	0.00388^*∗∗∗*^
	(0.00662)	(0.00633)	(0.00833)	(0.00127)
ICT social impact	−0.0147^*∗*^	−0.0116	−0.0169^*∗*^	0.000749
	(0.00759)	(0.00727)	(0.00958)	(0.00146)
GDP	−0.412^*∗∗∗*^	−0.336^*∗∗∗*^	−0.220^*∗∗∗*^	0.0843^*∗∗∗*^
	(0.0347)	(0.0333)	(0.0438)	(0.00666)
Constant	13.55^*∗∗∗*^	11.44^*∗∗∗*^	9.334^*∗∗∗*^	2.145^*∗∗∗*^
	(0.846)	(0.810)	(1.066)	(0.162)
Observations	660	660	662	662
R-squared	0.629	0.620	0.368	0.438
Number of id	140	140	141	141

Standard errors in parentheses ^*∗∗∗*^*p* < 0.01, ^*∗∗*^*p* < 0.05, ^*∗*^*p* < 0.1

**Table 7:** Mediated effect result overview.

Dependent variables	Under-five mortality rate		Adolescent fertility rate	
Mediating variables	ICT social impact		ICT social impact	
Independent variables	ICT environment	ICT usage	ICT environment	ICT usage
Sobel Z	−1.801	−1.855	−1.654	−1.695
Sobel *p* value	0.07163448	0.06357	0.09814432	0.09001181
Goodman-1 Z	−1.769	−1.834	−1.624	−1.676
Goodman-1 *p* value	0.07687708	0.06662993	0.10447248	0.09375428
Goodman-2 Z	−1.836	−1.877	−1.686	−1.715
Goodman-2 *p* value	0.06641567	0.06052563	0.09178463	0.08626387
Proportion of total effect that is mediated	0.09574541	0.0518865	0.09248442	0.07066528

**Table 8:** Results of hypothesis testing.

Hypothesis	Result
H1	Partially supported
H2	Partially supported
H3	Partially supported
H4	Partially supported
H5	Partially supported

## Data Availability

All the data used in our study could be approached upon request.
